The article "Effect of WeChat-Based Health Education Combined with Satir Model on Self-Management Behaviors and Social Adaptation in Colorectal Cancer Patients during the Perioperative Period" was published in 2021. Journal: J Healthc Eng.

# Effect of WeChat-Based Health Education Combined with Satir Model on Self-Management Behaviors and Social Adaptation in Colorectal Cancer Patients during the Perioperative Period

**DOI:** 10.1155/2021/2701039

**Published:** 2021-12-10

**Authors:** Limin Feng, Weina Wang, Meiying Wu, Huili Ma

**Affiliations:** ^1^Department of Gastrointestinal Surgery, Yantai Yuhuangding Hospital, Yantai 264000, Shandong Province, China; ^2^Department of Surgical Care, Rizhao Hospital of Traditional Chinese Medicine, Rizhao 276800, Shandong Province, China; ^3^Health Management Center, Qingdao Fuwai Cardiovascular Hospital, Qingdao 266011, Shandong Province, China; ^4^Department of Emergency Surgery, Binzhou Medical University Hospital, Binzhou 256603, Shandong Province, China

## Abstract

**Objective:**

To explore the effect of WeChat-based health education combined with the Satir model on self-management behaviors and social adaptation in colorectal cancer (CRC) patients during the perioperative period.

**Methods:**

A total of 100 CRC patients treated in our hospital from April 2018 to April 2020 were selected as the objects for the retrospective study and divided into the observation group and the reference group according to their admission order, with 50 cases each. The patients in both groups accepted health education based on the WeChat platform, and additionally, those in the observation group received the Satir group intervention on self-approval for 3 months to compare the patients' scores on self-management behaviors, social adaptation, and self-care agency before and after the intervention between the two groups.

**Results:**

Between the observation group and the reference group, the patients' general information, including age, gender ratio, and course of the disease, was not statistically different (*P* > 0.05). After nursing intervention, the scores on patients' self-management behaviors, social adaptation, and self-care agency were significantly higher in the observation group than in the reference group (*P* < 0.001).

**Conclusion:**

Combining the WeChat-based health education with the Satir model can improve the self-management awareness in the CRC patients during the perioperative period, enhance their self-care agency and self-management behaviors, and promote their social adaptation, demonstrating that such a nursing intervention model is worthy of clinical promotion.

## 1. Introduction

Colorectal cancer (CRC) originates from the epithelium of the large intestine, and it can be classified as colon cancer and rectal cancer. The most common pathological type of CRC is adenocarcinoma, while squamous cell carcinoma is a rare type [1, 2]. Globally, colorectal cancer incidences rank third in malignancy, and their mortality ranks second in malignancy-related deaths [3]. The data from the World Health Organization study showed that there were 1.8 million new colorectal cancer cases and 88,000 deaths from the disease worldwide in 2018, indicating that 1 patient was diagnosed every 3.5 min and 1 patient died of colorectal cancer every 9 min [4, 5]. Because of the deep and low position of colorectal cancer lesions in the pelvic cavity, a colostomy is mainly applied to patients at the present stage [6]. A colostomy is defined as creating a permanent artificial anus for the patients with surgery, which can effectively improve their symptoms. However, it will change their normal bowel movements, and it is associated with many postoperative complications, such as injurious dermatitis, canal prolapse, and parastomal hernia, causing serious preoperative resistance that is not conducive to surgery. Scholars Austin George et al., found that health education can reduce the perioperative anxiety of patients before surgery and reduce their psychological stress, which is good for enhancing the perioperative nursing outcomes [7]. Information-based nursing has now become an important trend in the development of the nursing field, and hence, health education shall also be based on informatization to fully enhance its efficiency [8]. WeChat is the most commonly used communication software for Chinese residents. It is free of charge, works in real time, and is easy to operate. The study by Zhang et al. has confirmed that WeChat is a good tool to improve the health knowledge level of patients and that it is beneficial for enhancing the perioperative nursing management of the nursing personnel [9, 10].

For surgical CRP patients, the lack of relevant knowledge and changes in their self-image cause negative emotions in the perioperative period [11]. They often have a sense of shame because of the intestinal stoma, and their social interaction and daily life are significantly affected in a negative way. Hence, they are prone to postoperative anxiety and depression and even develop mental illness in severe cases, which affects the recovery process. Although carrying out health education with WeChat can promote the perioperative cooperation of patients, it cannot improve their psychological condition, and therefore, they still have poor social adaptation, lower self-management ability, and difficulty in returning to normal life. In recent years, people's perception of mental state in patients with malignant tumors has continued to deepen, and some studies have found that group intervention enables the patients to gain a sense of identity and alleviates their psychological repellence [12]. The Satir model is an intervention model centered on humanism, which aims to promote the patients' dignity, help them accept themselves, and achieve physical and mental harmony. Currently, the Satir model is less used in the nursing of malignant tumors. It is a novel intervention mode, especially for CRC patients. Hence, its application effects need further exploration. Based on this, health education with WeChat was combined with the Satir model herein to explore which nursing mode had an actual effect on surgical CRC patients, with the results summarized as follows:

## 2. Data and Methods

### 2.1. Study Design

The study was conducted in our hospital from April 2018 to April 2020 to explore the effect of combining WeChat-based health education with the Satir model on self-management behaviors and social adaptation in CRC patients during the perioperative period. It was a retrospective study, and the blind level was double-blind.

### 2.2. Study Object Enrolment

Inclusion criteria: (1) the patients were diagnosed with colon cancer or rectal cancer after the pathological and imaging examinations and accepted a colostomy for the first time [13], (2) the patients were treated in our hospital during the whole course and had complete clinical data, (3) the estimated survival of the patients was more than 6 months, (4) the patients had normal cognitive ability and were able to use WeChat or had the ability of learning to use WeChat, (5) the patients were at least 18 years old, and (6) the patients did not have postoperative tumor metastasis, relapse, etc.

Exclusion criteria: (1) the patients had other malignant tumors, (2) the patients had immune diseases, (3) the patients had inflammatory diseases, (4) the patients had mental problems and could not communicate with others, (5) the patients had congenital abnormalities, (6) the patients could not take care of themselves in daily life, (7) the patients had severe postoperative complications, and (8) the patients had remote metastasis of tumor.

### 2.3. Study Object Grouping

A total of 100 CRC patients treated in our hospital from April 2018 to April 2020 were selected as the study objects and divided into the observation group and reference group according to their admission order, with 50 cases each. The patients' general information was not statistically different between the two groups (*P* > 0.05), and hence, the patients could be selected as the study objects. See Table 1.

### 2.4. Moral Standard

The study met the principles in *World Medical Association Declaration of Helsinki (2013)* [14], and all patients and their family members signed the informed consent.

### 2.5. Study Methods

The patients in both groups accepted WeChat-based health education with specific steps. (1) A WeChat health education group was set up, and the group members included the head nurse and nursing personnel who had working experience in the oncology department and professional knowledge. By adopting evidence-based nursing and combining it with the working experience in the hospital, the group members reviewed a great deal of information about the health education of CRC in the perioperative period and formulated a corresponding education framework. (2) The group members shared the work, cooperated with one another, and implemented the policy of individual responsibility. The nursing personnel established the information base of the patients for whom they were responsible and invited them to the WeChat group. The health record should include the patients' name, gender, age, marital status, educational degree, occupation, income level, payment method of medical fees, drinking history, smoking history, disease site, and pathological stage. (3) One nurse compiled the WeChat push message on general health education, and other nurses compiled the personalized messages according to the recovery status of patients, mainly including relevant disease knowledge, personalized diet and schedule, medication dosage, maintenance of deep venous catheter, and familial self-care. (4) The WeChat push message on health education should be sent out of the normal rest time. The time for sending the public message should be between 7 : 00 pm and 8 : 00 pm, and the time for sending the personal message should be between 8 : 00 pm and 9 : 00 pm. The frequency of sending the messages should be 3 times per week for 1 month before surgery and 2 months after surgery. (5) After sending the message, the nursing personnel should ask for patient feedback, interact with the patients, and answer their questions and doubts. For the patients who did not reply, the nursing personnel could ask the patients face-to-face about the reasons for not replying and call the patients via telephone after discharge to improve the patients' degree of recognition of WeChat health education.

On this basis, the patients in the observation group received the Satir group intervention on self-approval with specific steps. (1) The WeChat health education group was also the Satir intervention group with another 2 psychologists included. The psychologists conducted professional knowledge training to the nursing personnel, established the Satir group intervention plan on self-approval, and selected the activity site for group intervention 2 times per week for 3 months. (2) Firstly, the group members enlivened the atmosphere of the WeChat group, encouraged the patients to speak and gained their trust, and invited them to join the group intervention. At patients' first intervention, small games were played to help them introduce themselves and create an open, easy, and active environment so that the patients gradually relaxed and established a trusting relationship. (3) The postoperative well-recovered patients were invited to give speeches so that other patients could reshape their confidence and understand themselves. The group members, successful cases, and enrolled patients communicated with each other face-to-face about the impact of surgery and discussed the postoperative self-changes together. The nursing personnel listened to the patients carefully, encouraged them actively to open up and share their vision, and helped them find a suitable and feasible living style and face the life challenges after surgery. (4) During the activity, the nursing personnel used more inspiring words to guide the patients on self-care and improve their self-care agency, such as relieving negative emotions by means of abdominal breathing and meditation. At the same time, the patients' family members learned the nursing methods for intestinal stomas, and for those with lower familial nursing ability, one-on-one training was carried out to inform them of the usage of the leak-proof cream and correctly recognize the complications, such as stoma edema. They were advised to think from the perspective of patients and provide family support. (5) The nursing personnel should help patients with self-esteem building and gently tell them that the stoma was a part of the body that required recognition and care so that the patients would not deny their value because of cancer, restart their hobbies, and increase their sense of self-worth.

### 2.6. Observation Criteria

1. General information: It included gender, age, postoperative pathological stage, education background, marital status, stoma type, course of disease, and payment method of medical fees.
2. Scores on self-management behaviors: The patients' self-management behaviors before and after the nursing intervention were evaluated with the Self-management Behaviors Scale [15] compiled by Li Hui, which was applicable to CRC patients with its credibility proven by domestic literature. The scale contained 4 dimensions, namely, partnerships, problem-solving, the execution of self-management, and emotion handling, along with 20 items. On a scale of 0–80 points, the higher scores indicated better self-management behaviors.
3. Scores on social adaptation: The patients' social adaptation before and after the nursing intervention was evaluated based on the Ostomy Social Mentality Adjustment Scale [16] revised by Xu Qin et al., which was applicable to CRC patients with its credibility proven by domestic literature. The scale contained 3 dimensions, namely, positive emotions, negative emotions, and social life adaptation, along with 20 items. On a scale of 0–80 points, the higher scores indicated a stronger social adaptation.
4. Scores on self-care agency: The patients' self-care agency before and after the nursing intervention was evaluated based on the Exercise of Self-Care Agency (ESCA) [17] scale complied by Keamey and Fleischer whose credibility and effectiveness are proved by domestic and foreign literature. The scale contained 4 dimensions, namely, self-concept, health knowledge level, self-care agency, and responsibility for self-care, along with 43 items. On a scale of 0–127 points, the higher scores indicated a better self-care agency.

### 2.7. Statistical Processing

In this study, the data processing software was SPSS20.0, the picture drawing software was GraphPad Prism 7 (GraphPad Software, San Diego, USA), the enumeration data were examined by X2 test, the measurement data were examined by *t*-test, and the differences were considered statistically significant at *P* < 0.05.

## 3. Results

### 3.1. Comparison of Patients' General Information

The patients' general information, including age, gender ratio, and course of disease, were not statistically different between the observation group and the reference group (*P* > 0.05). See Table 1.

### 3.2. Comparison of Scores on Patients' Self-Management Behaviors

After the nursing intervention, the scores on self-management behaviors were significantly higher in the observation group than in the reference group (*P* < 0.001). See Figure 1.

In Figures 1(a) and 1(b), the horizontal axes from left to right indicated partnerships, problem-solving, the execution of self-management, and emotion-handling. The vertical axes indicated the self-management behavior score (points). The black areas indicated the observation group, the gray areas indicated the reference group, and # indicated *P* < 0.001.

Figure 1(a) shows the scores on self-management behaviors before the nursing intervention of the two groups, and between the observation group and the reference group, the scores on partnerships (12.11 ± 0.98 vs 12.14 ± 0.96), problem-solving (13.11 ± 0.68 vs 13.09 ± 0.70), the execution of self-management (17.64 ± 0.80 vs 17.68 ± 0.75), and emotion-handling (8.11 ± 0.45 vs 8.10 ± 0.52) were not statistically different (*P* > 0.05).

Figure 1(b) shows the scores on self-management behaviors after the nursing intervention of the two groups, and between the observation group and the reference group, the scores on partnerships (17.45 ± 0.68 vs 14.99 ± 0.87), problem-solving (20.11 ± 0.87 vs 17.24 ± 0.68), the execution of self-management (25.14 ± 0.78 vs 23.10 ± 0.99), and emotion-handling (13.99 ± 0.45 vs 11.65 ± 0.54) were significantly higher in the observation group than in the reference group (*P* < 0.001).

### 3.3. Comparison of Scores on Patients' Social Adaptation

After the nursing intervention, the scores on social adaptation were significantly higher in the observation group than in the reference group (*P* < 0.001). See Figure 2.

In Figures 2(a) and 2(b), the horizontal axes from left to right indicated positive emotions, negative emotions, and social life adaptation, whereas the vertical axes indicated the social adaptation score (points). The black areas indicated the observation group, the gray areas indicated the reference group, and # indicated *P* < 0.001.

Figure 2(a) shows the scores on social adaptation before the nursing intervention of the two groups, and between the observation group and the reference group, the scores on positive emotions (17.10 ± 1.23 vs 17.05 ± 1.11), negative emotions (12.65 ± 0.98 vs 12.71 ± 0.86), and social life adaptation (21.65 ± 2.68 vs 21.70 ± 2.40) were not statistically different (*P* > 0.05).

Figure 2(b) shows the scores on social adaptation after the nursing intervention of the two groups, and between the observation group and the reference group, the scores on positive emotions (22.65 ± 2.20 vs 19.98 ± 1.68), negative emotions (22.51 ± 2.35 vs 19.10 ± 1.98), and social life adaptation (29.12 ± 3.65 vs 22.15 ± 2.65) were significantly higher in the observation group than in the reference group (*P* < 0.001).

### 3.4. Comparison of Scores on Patients' Self-Care Agency

After the nursing intervention, the scores on self-care agency were significantly higher in the observation group than in the reference group (*P* < 0.001). See Figure 3.

In Figures 3(a) and 3(b), the horizontal axes from left to right indicated self-concept, health knowledge level, self-care ability, and responsibility for self-care, whereas the vertical axes indicated the self-care agency score (points). The black areas indicated the observation group, the gray areas indicated the reference group, and # indicated *P* < 0.001.

Figure 3(a) shows the scores on self-care agency before the nursing intervention of the two groups, and between the observation group and the reference group, the scores on self-concept (20.15 ± 1.68 vs 20.25 ± 1.70), health knowledge level (19.98 ± 1.22 vs 19.95 ± 1.34), self-care ability (19.10 ± 1.22 vs 19.12 ± 1.20), and responsibility for self-care (19.98 ± 1.20 vs 20.01 ± 1.23) were not statistically different (*P* > 0.05).

Figure 3(b) shows the scores on self-care agency after the nursing intervention of the two groups, and between the observation group and the reference group, the scores on self-concept (31.22 ± 2.68 vs 25.41 ± 2.65), health knowledge level (31.55 ± 3.21 vs 25.98 ± 2.65), self-care ability (32.98 ± 3.65 vs 22.10 ± 1.68), and responsibility for self-care (29.98 ± 2.98 vs 22.10 ± 2.15) were significantly higher in the observation group than in the control group (*P* < 0.001).

## 4. Discussion

At present, a permanent colostomy is the main treatment method for CRC. However, the changes in the physiological structure because of surgery can cause various types of psychological problems in patients. They mainly manifest as anxiety, resistance, fear, negative coping, and reluctance to cooperate with clinical treatment and nursing before surgery. After surgery, they may manifest as depression, sensitivity, declined self-management ability, and poor social adaptation, thus reducing the surgery's effect and the patients' willingness to return to society, which, in part, deviates from the central significance of malignant cancer treatment. As people's perspective on patients with malignant tumors has changed, prolonging the life span is no longer the only purpose of cancer treatment, while paying much attention to patients on the basis of protecting their life and health for them to regain dignity and meaningful life is the value of medical treatment [18, 19]. Currently, routine nursing is still the prevailing nursing model that aims to prolong the survival of patients with malignant tumors. However, it lacks personalized psychological interventions and cannot sufficiently improve the psychological condition of patients. Domestic and foreign reports have shown that psychological and mental conditions are an important factor affecting the treatment effect of patients, and strengthening the psychological intervention can not only meet the demand of modern human standard nursing but also further enhance the treatment effect of patients and improve their self-management ability [20, 21].

The Satir model is a type of humanist-based intervention therapy developed by the American scholar Virginia Satir. It focuses the intervention content on individual self-esteem that involves selfhood, others, situations, etc., with the aim of helping individuals in achieving physical and mental harmony [22]. For surgical CRC patients, the Satir model is an effective tool for them to face their physiological changes, and its positive meaning lies in that the patients can deeply feel that they are not alone in fighting the disease and that there are many people facing the same situation, thereby alleviating their loneliness and inferiority feeling. In addition, compared to the conventional psychological intervention, the Satir model improves the patients' trust [23]. To be specific, in a relaxed and loving group atmosphere, the patients can gradually build a sense of communication and trust to share their own experiences with those undergoing the same situation and benefit from the positive experiences of others. Therefore, the study results showed that the negative emotions in the patients of the two groups were relieved, and their positive emotions were increased, indicating that the group effect worked well in promoting social adaptation.

Under the premises of all patients receiving WeChat health education, the social adaptation of patients in the observation group was stronger. It was because of the fact that although WeChat health education could objectively enhance the patients' health knowledge levels, their self-care ability, responsibility for self-care, and the execution of self-care still depended on their psychological and mental conditions. If patients have impaired self-esteem and faulty self-value perceptions, their enthusiasm to perform self-care decreases, which may not be improved even with the health education. Hence, the key to exerting the effect of health education still lies in regulating and improving the patients' self-perception. During the course of carrying out the Satir group intervention, the nursing personnel should pay attention to respecting the value of the patient as an individual, fully affirming their meaning of survival so that the patients can once again feel the dignity of life [24]. Scholars Daniels et al. reported that exploring the value of life with patients suffering from malignant tumors through praise and encouragement enables them to regain life faith and reduce the willingness to commit suicide [25]. The study found that after the nursing intervention, scores on patients' self-management behaviors and self-care agency were significantly higher in the observation group than in the reference group (*P* < 0.001), indicating that the people-oriented Satir model could make the patients recognize again their own value and enhance the enthusiasm of self-management.

In conclusion, combining WeChat-based health education with the Satir model can improve self-management behaviors and social adaptation in CRC patients during the perioperative period. It presents good social value, and hence, it should be promoted in practice.

## Figures and Tables

**Figure 1:** Comparison of scores on patients' self-management behaviors ($\bar{x}$ ± *s*, points).

**Figure 2:** Comparison of scores on patients' social adaptation ($\bar{x}$ ± *s*, points).

**Figure 3:** Comparison of scores on patients' self-care agency ($\bar{x}$ ± *s*, points).

**Table 1:** Comparison of patients' general information.

Group	Observation (*n* = 50)	Reference (*n* = 50)	X^2^/*t*	*P*
**Gender**			0.041	0.840
**Male**	28	29		
**Female**	22	21		
**Age (years)**				
**Range**	25–76	28–72		
**Mean age**	49.98 ± 2.65	50.22 ± 2.98	0.426	0.671
**Postoperative pathological stage**				
**I**	20	22	0.164	0.685
**II**	18	15	0.407	0.523
**III**	12	13	0.053	0.817
**Educational background**				
**Primary school and below**	8	6	0.332	0.564
**Technical secondary school**	22	24	0.161	0.688
**Junior college and above**	20	20	0.000	1.000
**Marital status**			0.457	0.499
**Married**	35	38		
**Unmarried (widowed)**	15	12		
**Course of disease (months)**	8.00 ± 0.65	8.05 ± 0.58	0.405	0.686
**Stoma type**			0.191	0.663
**Sigmoid colon**	34	36		
**Transverse colon**	16	14		
**Payment method of medical fees**				
**Medical insurance**	18	20	0.170	0.680
**Commercial insurance**	15	15	0.000	1.000
**New rural cooperative medical insurance**	8	6	0.332	0.564
**Others**	9	9	0.000	1.000

## Data Availability

The data supporting the findings of this study are available on reasonable request from the corresponding author.
